This article has been retracted.

# Exemestane blocks mesothelioma growth through downregulation of cAMP, pCREB and CD44 implicating new treatment option in patients affected by this disease

**DOI:** 10.1186/1476-4598-13-69

**Published:** 2014-03-21

**Authors:** Barbara Nuvoli, Sabrina Germoni, Carlotta Morosetti, Raffaela Santoro, Giancarlo Cortese, Serena Masi, Iole Cordone, Rossella Galati

**Affiliations:** 1 Molecular Medicine Area, Regina Elena National Cancer Institute, Rome 00144, Italy; 2 S.A.F.U. Department, Regina Elena National Cancer Institute, Rome, Italy; 3 Clinical Pathology, Regina Elena National Cancer Institute, Rome, Italy

**Keywords:** Mesothelioma, Aromatase, Exemestane

## Abstract

**Background:**

Recent evidence suggests that aromatase may be involved in the pathogenesis of malignant mesothelioma. Here, we evaluated the effect of exemestane, an inhibitor of aromatase, in the treatment of mesothelioma using *in vitro* and *in vivo* preclinical models.

**Results:**

We show a significant reduction of cell proliferation, survival, migration and block of cells in S phase of cell cycle in mesothelioma cells upon exemestane treatment. Moreover, we find that CD44, which is involved in mesothelioma cells migration, was modulated by exemestane via cAMP and pCREB. Most importantly, in mice mesothelioma xenograft exemestane causes a significant decrease in tumor size and the association pemetrexed/exemestane is more effective than pemetrexed/cisplatin.

**Conclusion:**

The preclinical mesothelioma model suggests that exemestane might be beneficial in mesothelioma treatment.

## Background

Malignant Mesotheliomas (MM) are aggressive and lethal neoplasms arising from mesothelial cells lining the pleura, peritoneum, tunica vaginalis testis and pericardium. Human malignant pleural mesothelioma (MPM) is the most common form of mesothelioma that grows aggressively, with dissemination throughout the pleural cavity, and is frequently associated with massive pleural effusion [1]. MPM is considered to be closely associated with a personal history of prolonged exposure to asbestos fibres in patients [2,3], although several etiologic factors iron [4] and simian virus 40 (SV40) [5] are reported to be involved in the development of MPM. The incidence of MPM is expected to increase at an alarming rate over the next few years, despite the banning of asbestos. Disease incidence varies markedly within and between countries. The highest annual rates of disease, approximately 30 case per million, are reported in Australia and Great Britain. The risk of disease increases with age and is higher in men. Time from asbestos exposure to disease diagnosis is on average greater than 40 years. Non occupational asbestos exposures contribute an increasing proportion of disease. With the exception of the United States, incidence continues to be on the increase. In developed countries peak incidence is expected to occur before 2030 [6,7]. MPM, sometimes takes 10 years or more for changes to appear that are indicative of pleural disease, and even longer for symptoms to manifest. Patients frequently present respiratory symptoms, including dyspnea, shortness of breath and chest pain, extremely limiting the quality of life of the patients with this disease. Following diagnosis, most cases of malignant mesothelioma have poor survival [1]. The standard therapeutic modalities for MPM, including surgery, chemotherapy and radiation, have yielded unsatisfactory outcomes [8]. The combination of cisplatin and pemetrexed has become standard first-line therapy worldwide for patients who are not suitable for aggressive surgery, or in whom chemotherapy is recommended as part of a multimodality regimen with a mean survival of 12.1 months and 18.34 [9-11]. Therefore, in order to improve the clinical outcome in the pharmacological treatment of this refractory tumour, drugs aimed at targeting novel and/or characterized tumour-specific cellular targets are needed. The pathogenic mechanisms underlying mesothelioma involve epigenetic gene regulation [12] and deregulation of multiple signaling pathways, including sonic hedgehog signalling [13,14], activation of multiple receptor tyrosine kinases such as the epidermal growth factor receptor (EGFR) family and MET, and subsequent deregulations of mitogen-activated protein kinase (MAPK) and phosphatidylinositol-3-kinase (PI3K)-AKT signaling cascades, the TNF-α/NF-κB survival pathway, Wnt signaling, and loss of tumor suppressors such as Neurofibromatosis type 2, p16INK4A, and p14ARF [15,16]. Understanding the mechanisms of the dysregulated signaling pathways allows strategies for development of targeted new therapies against this devastating disease.

Recently, we have demonstrated the presence of aromatase (CYP19A1) in MPM cell lines and tumor tissue sections from patients with MPM [17,18]. CYP19A1 was expressed in the majority of MPM samples as a cytoplasmic protein and the cytoplasmic expression of CYP19A1 significantly correlated with poor survival [17]. The World Health Organization classifies MM into epithelial, sarcomatoid, and biphasic types, each of which can be subdivided further. This classification has implications for both diagnosis and prognosis [19]. Prognosis is poor for all MMs, but sarcomatoid MMs have a particularly poor response rate to treatment: a significant association between high expression of CYP19A1 and sarcomatoid MPMs was found [17]. These observations suggested that CYP19A1 plays a role in tumour progression in MPM. CYP19A1 is a key enzyme in the biosynthesis of estrogen (converting testosterone into estradiol (E2). Females were identified as being a positive prognostic factor for peritoneal MM: female patients have a median survival than males (17.3 months compared to 11.8 months respectively) [20,21]. The estrogen receptors expression using immunohistochemistry, was demonstrated in peritoneal tumors and not in pleural tumors [22]. Recently, immunohistochemical analysis revealed intense nuclear ERβ staining in normal pleura that was reduced in MM tissues. Conversely, neither MM nor normal pleura stained positive for ERα [23]. This leads to more carefully explore the role of estrogen in the pathogenesis of MM and especially on MPM.

Exemestane an inhibitor of CYP19A1 type 1 (steroidal inactivator), induces cell death in Ist Mes1, Ist Mes2 and MPP89 MPM cell lines [17]. This initial finding has provided the impetus for the studies presented here, aimed to investigate the mechanism of action of exemestane on MPM cells and xenograft MPM models. We have thus identified possible pathways between cyclic adenosine monophosphate (cAMP), cAMP response element-binding protein (CREB), CD44 and pAKT, Bcl-xL that are downregulated by exemestane in MPM cells sensitive. Finally, we demonstrated that exemestane was effective *in vivo* alone and in combination with pemetrexed, and that the effect of this association was superior compared to the therapeutic combination cisplatin/pemetrexed.

## Results

### Exemestane inhibits MPM cell growth *in vitro*

Exemestane was used to evaluate the impact of CYP19A1 blockade in our MPM preclinical models. Met-5A, MSTO and NCI cells were treated with incremental drug doses for 24 and 48 hours. Exemestane 35 and 70 μM induced a significant (P < 0.05) dose-dependent decrease of metabolic activity in MSTO (Figure 1A). Only with exemestane 70 μM at 48 h a significant (P = 0.0036) reduction of the metabolic activity in NCI was observed (Figure 1A). Exemestane 35 and 70 μM was no active in Met-5A (Figure 1B). Exemestane had antiproliferative action dose response dependent in MSTO (Figure 1C). For subsequent experiments, in an attempt to find the cause of the different levels of sensitivity to the drug between MSTO and NCI, the concentration of 35 μM that is closest to 50% of MSTO cell death and had no effect on NCI was chosen. Exemestane 35 μM reduced the colony formation capacity of MSTO whereas no difference compared to the control was observed in NCI and Met-5A (Figure 1D). Next, the effects of CYP19A1 inhibition on cell-cycle progression and apoptosis were evaluated. Upon 24 h exemestane treatment MSTO resulted in a cell cycle arrest in S-phase (Figure 1E). This was transient, as we could not observe 48 h post-treatment, probably due to its half-life. In agreement, increased levels of p21 and decreased Bcl-2 and Bcl-xL (Figure 1F) were detected in western blot. The effect of exemestane on MPM cell migration was evaluated. In MSTO and other exemestane sensitive MPM cell lines (Ist Mes1, Ist Mes2 and MPP89), the drug blocks migration (Figure 1G). Altogether, these results suggest that CYP19A1 blockade results in decreased MPM cell proliferation, S cell-cycle arrest and abrogation of the ability to migrate.

**Figure 1:** **Exemestane acts on MPM cell growth, cell-cycle progression and migration. A**, NCI was not very sensitive to exemestane (EXE), only 70 μM of drug for 48 h had a significant response versus untreated (CNTR) cells; **B**, exemestane was not effective in Met-5A. Significant decrease in MSTO cell growth was observed upon different exemestane dosage treatment as per XTT **(A)**, manual cell counting **(C)** and clonogenicity assays (35 μM exemestane) **(D)**. **E**, exemestane (35 μM) induced cell cycle arrest in S-phase; **F**, Western blotting showed increase in p21 and decrease in Bcl-2 and Bcl-xL expression. **G**, reduced MPM cell lines sensitive migration in response to 35 μM exemestane treatment was identified by wound healing assay. Cell migration was not inhibited in NCI. Graphs represent the average of at least 3 repeated experiments; *, statistically significant effects (P < 0.05).

### cAMP and CD44 are the targets of exemestane in MPM cell

We sought to identify the possible target of exemestane in MPM cell lines. Reports in the literature on other types of cancer cells indicate drug action on cAMP [24] and the involvement of CD44 in the migration of MPM cells [25]. As depicted in Figure 2A, MSTO, Ist-Mes1, Ist-Mes2 and MPP89 upon 30 min exemestane treatment exhibited decreased levels of cAMP levels, contrary to what happens to the NCI. This suggests that exemestane acts by modulating cAMP levels.

**Figure 2:** **Exemestane acts in MPM cells by cAMP and CD44. A**, cAMP ELISA detects a decrease in cAMP levels upon 35 μM exemestane treatment for 30 min (EXE), compared to untreated (CNTR), in all lines except NCI. **B**, western blot identifies CREB phosphorylation (pCREB) inhibition in cell lines responsive to exemestane treatment (E30) versus untreated (C30). **C**, flow cytometric characterizzazion of CD44 expression in untreated and treated MPM cell lines. Data are presented as a count of positive cells and numerical value indicates CD44 mean fluorescence intensity (MIF) of total cell population in the sample analyzed. Excluding NCI, all MPM cell lines show a reduction of MIF. **D**, siRNACD44 in MSTO and NCI reduced MPM cell lines migration in wound healing assay **E**, siRNA CD44 transfection resulted in decreased cell viability in MSTO and NCI cell lines compared to no CD44 siRNA. In addition, exemestane treatment further reduces the MSTO cell survival. No effect was observed in NCI. **F**, Western blot shows the silencing of CD44 occurring in MSTO and NCI. Moreover, the effect of exemestane in MSTO resulted in a decreased phosphorylation of AKT and CREB and in the reduction of Bcl-xL both in silenced cells that did not. No change was observed in NCI upon exemestane treatment both in silenced cells that did not. Graphs represent the average of at least 3 repeated experiments; *, statistically significant effects (P < 0.05).

Western blott analysis shown an involvement of pCREB in drug action (Figure 2B) and a direct correlation between cAMP level and pCREB expression was observed. No change in total CREB was detected. Based on what we postulate, pCREB was activated by cAMP also in MPM.

FITC-CD44 analysis, by flow cytometry, shows a reduction of fluorescence only in cells sensitive to exemestane thus indicating that CD44 as a possible target of the drug (Figure 2C). To test this assumption, we silenced CD44 in MSTO and NCI and then investigated the effect on migration. The silencing of CD44 in MSTO and NCI inhibited the wound healing confirming the role of CD44 in cell migration (2D). Figure 2E shows the mean relative viabilities of MSTO and NCI cells treated for 24 h with or without the CD44siRNA in the presence or absence of exemestane. It is evident that the silencing of CD44 kills both cell lines, consequently, we can deduce that CD44 was essential in the cellular growth. Moreover, the siRNACD44 does not make MPM cell lines more sensitive to the action of the drug. Thus, suggesting that in both cell lines, the direct target of exemestane might be some factor upstream of CD44 that in NCI was not a target upon 35 μM exemestane treatment. MSTO and NCI without and with CD44si RNA show the same pattern of pCREB and pAKT (Figure 2F MSTO Lane1,3; NCI Lane5,7) and total AKT and CREB (data not show). Exemestane decreases pAKT, pCREB and Bcl-xL in MSTO (Figure 2F Lane 2,4) and not total AKT and CREB. In contrast, no change was observed in NCI pointing out pAKT, pCREB and Bcl-xL as possible targets of the drug (Figure 2F Lane 5,7).

### Exemestane inhibits MPM cell growth *in vivo*

We next sought to evaluate whether the antiproliferative effect of exemestane can also be observed *in vivo*. Using a MPM xenograft animal model resulting from the subcutaneous injection of MSTO cells, we compared the effect of exemestane alone or in association with pemetrexed on tumor growth in immunodeficient mice as compared to administration of the control vehicle (physiological solution) and cisplatinum pemetrexed respectively (Figure 3). We decided not to include in the study groups of mice treated with cisplatinum or pemetrexed alone because the purpose was to assess whether the exemestane-pemetrexed combination was more effective than standard therapy.

**Figure 3:** **Exemestane alone and in association with pemetrexed blocks growth of MPM tumor xenografts. A**, Graphs represent 100 days of tumor volume measurements in mice treated (EXE) or not (CNTRL) with exemestane for 60 days. **B**, Graphs represent 100 days of tumor volume measurements in mice upon cisplatin-pemetrexed (C-P) or exemestane-pemetrexed (E-P) treatment for 60 days versus non treated mice (CNTRL). Each value represents the average and standard deviation, P is the p value assessed using 2-tailed Student’s test.

Since exemestane is a drug implicated in estrogen synthesis, we used in the *in vivo* experiments mixed sex mice (5 male and 5 female) for each group of treatment. The treatment with exemestane for 60 days induced a significant reduction (p = 0.03) of tumor growth compared to the control group in 40 days. During therapy and for 40 days after the end of treatment the mice were in good health and the tumor continued to decline significantly (p = 1.2 × 10^-5^) until the complete healing of 9 out of 12 mice in 100 days (Figure 3A). The association cisplatin-pemetrexed and exemestane-pemetrexed were significantly effective versus CNTRL with a p value of 5.2 × 10^-4^ and 1.8 × 10^-5^ respectively already in 30 days of treatment. At same time, the association exemestane-pemetrexed was significantly (P = 3.3 × 10^-4^) more effective than cisplatin-pemetrexed (Figure 3B). 40 days after the end of treatments, 3 mice treated with cisplatin-pemetrexed were dead and only 1 showed a complete reduction in the mass, while in mice treated with exemestane-pemetrexed 1 was dead and 7 showed a complete reduction of the mass. The deviation standard in Figure 3, especially at 100 days time point is very high because it takes into accountb both the mice in which the tumor has disappeared and not. These data support the use of exemestane in the care of MPM.

## Discussion

The current study highlights the effect of exemestane and its potential translation into the clinical setting for the treatment of MPM. A recent study reported the presence of CYP19A1 in cells and tissues of MPM and the antiproliferative action of exemestane in Ist-Mes1, Ist-Mes2 and MPP89 [17]. Normal mesothelium exhibited a weak positivity for CYP19A1 and the human pleuralmesothelial cell Met-5A does not express appreciable levels of CYP19A1 by western blot. Met-5A was not sensitive to exemestame treatment. In order to better understand the mechanism of action of exemestane *in vitro* and *in vivo* we studied other two MPM cell lines, MSTO tumorigenic in mice and NCI. Exemestane 35 μM was found to inhibit the growth of MSTO cells *in vitro*, inducing arrested cell-cycle progression abrogated the tumor cell migration and reduced the colony formation capacity (Figure 1). On the contrary, nothing like what was observed in NCI, therefore this line was defined cell resistant to 35 μM of drug. *In vitro* experiments performed on MPM sensitive cell lines (MSTO, Ist-Mes1, Ist-Mes2 and MPP89) and NCI resistent cell lines upon exemestane treatment have helped us to identify drug targets. The exemestane dosage for all experiments was of 35 μM. Although the selected concentrations seem to be high, similar concentrations of an aromatase inhibitor have also been used in previous studies for *in vitro* experiments [24,26]. The dose of exemestane currently used in clinical practice is 25 mg daily. Exemestane exhibits an excellent safety profile in humans, having no significant toxicity at doses up to 600 mg/day and it is exceptionally well tolerated [27]. At clinically administered doses, the plasma half-lives of exemestane was 27 hours [28]. Exemestane is an irreversible, steroidal aromatase inactivator, structurally related to the natural substrate androstenedione. It acts as a false substrate for the aromatase enzyme and is processed to an intermediate that binds irreversibly to the active site of the enzyme causing its inactivation, an effect also known as “suicide inhibition” [29].

Another possible mechanism includes changes in aromatase activity through a cAMP-dependent mechanism [30]. A previous study reported an increase of cAMP levels in lung cancer cell lines, 15 min after treatment of cells with exemestane. This effect was reversed 30 min after the application of exemestane [24]. MPM cell lines sensitive upon 30 min exemestane treatment exhibited decreased levels of cAMP levels. This difference could be due to the different tissue types of origin. cAMP is a ubiquitous second messenger. Many growth factors and hormones regulate cellular activity through second messengers which correspondingly induce multifunctional protein kinases [31].

Activation of cAMP signaling involves binding of an extracellular ligand to a GPCR which through G proteins regulates one of several isoforms of adenylyl cyclase (AC) leading to cAMP generation. Although other effectors of cAMP have been identified, the most common downstream effector system is cAMP-dependent protein kinase (PKA). In its inactive state, the PKA holoenzyme consists of two catalytic (C) subunits bound noncovalently to a regulatory (R) subunit dimmer [32]. Binding of four cAMP molecules, two to each R subunit, leads to a conformational change and dissociation into an R subunit dimer with four cAMP molecules bound and two C monomers [33]. The C subunits then become catalytically active and phosphorylate serine and threonine residues on specific substrate proteins [34]. When cAMP rises, the C subunit released from the holoenzyme enters the nucleus by passive diffusion where it regulates a number of cellular processes, including motility, metabolism, neurotransmitter release, and transcription by the reversible phosphorylation of key substrates [35]. cAMP regulates the expression of specific genes by mediating the PKA-dependent phosphorylation of the CREB transcription factor in a 30-min period [31]. In MPM cell lines treated with exemestane, we found a direct correlation between levels of cAMP and expression of p-CREB. In particular the lines sensitive to exemestane treatment showed levels of cAMP and p-CREB decreased compared to controls untreated while in the line NCI resistant cAMP levels and p-CREB increased also in the presence of the drug (Figure 2A, B).

Exemestane inhibits cell migration in MPM cell lines sensitive to the agent. Data report CD44 responsible for cell migration in MM [25,36]. CD44 is a type I transmembrane glycoprotein (85–200 kDa) and functions as the major cellular adhesion molecule for hyaluronic acid, a component of the extracellular matrix. CD44 is expressed in most human cell types and is implicated in a wide variety of physiological and pathological processes, including lymphocyte homing and activation, cell migration, tumor cell growth, metastasis [37] and chemoresistance [38]. Flow cytometry (Figure 2C) revealed that MPM cell lines highly expressed CD44 and exemestane treatment reduces its levels in all lines except in NCI. The silencing of CD44 in MSTO and NCI confirms the importance of CD44 in cell migration and suggests its essential in the response to the drug, although the direct target of exemestane might be a factor upstream of CD44 that in NCI gives it resistance. Given the involvement of pAKT, Bcl-xL in Ist-Mes1, Ist-Mes2 and MPP89 drug response [17], we decided to assay their expression and p-CREB in CD44 silenced MSTO and NCI cells upon exemestane treatment and control. As shown in Figures 2E, p-CREB, pAKT and Bcl-xL expression were reduced by treatment with exemestane only in MSTO (silencied or not) indicating once again that the phosphorilation of these could be a target of the drug. Altogether, these data suggest that exemestane, reducing the levels of estradiol, affects cAMP and phosphoinositide 3-kinases (PI3K) pathway (Figure 4). Estrogen acts via the regulation of transcriptional processes, involving nuclear translocation and binding on specific response elements, thus leading to regulation of target gene expression. However, the observation of the effects induced by steroid hormones that are too fast to be mediated by the activation of RNA and proteins, has led to the identification of non- transcriptional mechanisms of signal transduction through steroid hormone receptors. These so-called “non-genomic” effects involve steroid-induced modulation of cytoplasmic or of cell membrane-bound regulatory proteins. Relevant biological actions of steroids have been associated with this signaling in different tissues. Ubiquitary regulatory cascades such as MAPK [39], the phosphatidylinositol 3-OH kinase (PI3K) and tyrosine kinases [40] are modulated through non-transcriptional mechanisms by steroid hormones. Steroid hormone modulation of cell membrane-associated molecules such as ion channels and G-protein-coupled receptors (GPCR) has been shown in diverse tissues [41]. Lines of evidence suggest that the estrogen-mediated activation of AC occurs independently of known ERs but rather requires GPR30 protein [42]. Since the exemestane induces a modulation of cAMP in short time (30 min) and considering that cAMP is produced upon AC activation, we ignored the classical estrogen receptors and focused on GPR30.

**Figure 4:** **Hypothesized mechanism of action of exemestane on MPM cells.** The GPCR receptor binds estrogen and cause estrogen-mediated cAMP stimulation and PI3K cascade. PI3K phosphorylates AKT (pAkt) which in turn regulates Bcl-xL, anti-apoptotic protein. cAMP stimulates PKA, which in turn activates CREB that translocates into the nucleus and acts as a transcription factor for CD44. The action of exemestane is carried out by reducing the levels of estradiol, its binding with GPCR and related downstream pathway.

The GPR30 receptor binds estrogen and cause estrogen-mediated AC stimulation and PI3K cascade. PI3K are family of lipid kinases capable of phosphorylating the 3’OH of the inositol ring of phosphoinositides. They are responsible for coordinating a diverse range of cell functions including proliferation and cell survival. PI3K phosphorylates AKT (pAkt) which in turn regulates Bcl-xL, anti-apoptotic protein. The AC catalyzes the formation of cAMP which stimulates PKA which in turn activates CREB (pCREB). pCREB translocates into the nucleus and acts as a transcription factor for several genes including CD44. PI3K and cAMP pathways inhibition by exemestane causes pAKT, BclxL, pCREB and CD44 down-regulation in MPM cell resulting in cell death. Intuitively, it can be hypothesized that the action of exemestane is achieved by reducing the levels of estradiol, its binding with GPR30 and related downstream pathway (Figure 4). Further studies are underway to validate the role of GPR30 in MPM. Using a MPM xenograft animal model resulting from the subcutaneous injection of MSTO cells, we compared the effect of exemestane on tumor growth in immunodeficient mice versus to control. Therapy was initiated after tumor establishment. Mice in both groups were followed for tumor size and toxicity. Treatment with exemestane induced tumor growth delay (Figure 3A) and decreased tumor mass completely in 70% of males and 80% of females as compared with control. Altogether, the impact of exemestane on MPM xenografts mirrors the effects noted in cell culture. Previous work shows the effectiveness of pemetrexed and cisplatin in MPM cell lines. Studies with the MSTO-211H cell line showed synergistic effects when pemetrexed was combined concurrently with cisplatin [43-45]. Pemetrexed is the first and only chemotherapy agent that has been granted marketing approval for use in combination with cisplatin for the treatment of chemonaive patients with unresectable MPM. Although pemetrexed combined with cisplatin showed a significant survival prolongation compared with cisplatin alone, the difference was only 2.8 months [46]. It is therefore necessary to augment the therapeutic effect of pemetrexed to further improve the survival of MPM patients. Therefore, given the growing body of clinical evidence suggesting only minimal effects of monotherapy, we decided to test the association exemestane-pemetrexed compared to standard combination cisplatin-pemetrexed in nude mice. Although the two treatments are effective in reducing the tumor mass, the association exemestane-pemetrexed was significantly (P = 0.039) more effective than cisplatin-pemetrexed (Figure 3B). In the present study, we clearly showed the increased efficacy of exemestane alone or in combination with pemetrexed versus the standard therapy pemetrexed-cisplatinum against MPM in the xenograft implantation model. In this context should not be underestimated that exemestane was as effective as the combination pemetrexed-exemestane, therefore exemestane monotherapy could be very beneficial to MPM patients.

We could not do a histologic examination to clarify the mechanism of the increased efficacy of exemestane and conventional chemotherapy because the therapy was so effective that we could not obtain enough tumor samples. These findings are encouraging and possibly support further investigation of exemestane in the clinical MPM context and highlight the opportunity to test, in the experimental MPM model, new compounds active with the same mechanism of action [47]. Exemestane is widely used in the treatment of breast cancer. It is active clinically in preventing, delaying progression of, and treating mammary cancers, many of which are estrogen receptor-positive. Exemestane 25 mg orally once daily was generally well tolerated without major toxicity [48] and it displays anti-inflammatory properties [49]. Given that exemestane has already been approved, it may proceed rapidly in clinical trials. After evaluating the benefits of exemestane alone or in association with chemotherapy in a group of patients, this therapy can be applied in MPM treatment protocols. Exemestane could possibly open new treatment strategies in association with standard therapy for patients afflicted with MPM. At present there are no clinical trials on the inhibitors of CYP19A1 in MPM, this may be probably due to the recent identification of CYP19A1 in MPM. In lung cancer, where studies of CYP19A1 are at a more advanced stage, some clinical studies consider the inhibitors of CYP19A1 an anti-oestrogen.

## Methods

### Cell lines and reagents

The human pleural mesothelial cell Met-5A and the human pleural MPM cell lines MSTO-211H (MSTO) and NCIH-2452 (NCI) were obtained from the American Type Culture Collection (ATCC) (Rockville, Md) and Ist-Mes1, Ist-Mes2, and MPP89 were obtained from Genova Institute Culture Collection. Cell lines were cultured as described previously [38]. Before treatment with exemestane, all cell lines were gradually conditioned in DMEM/F12 + Glutamax (Invitrogen) supplemented with 10% FBS and antibiotics.

The cell proliferation kit II (XTT) was purchased from Roche Molecular Biochemicals, Indianapolis, cAMP ELISA Kit from R&D Systems, the siRNA CD44 (5′GAACGAAUCCUGAAGACAU 3′, as 5′AUGUCUUCAGGAUUCGUUC3′) from Sigma, lipofectamine 2000 from Invitrogen, exemestane from Sequoia Research, Pemetrexed (Alimta) from Eli Lilly & Co, Cisplatino from Pfizer and Vitamina B12 (Dobetin) from Angelini SPA. Commercially available antibodies were used for immunoblo detection of: Bcl-2, p21, pCreb and CD44 (Santa Cruz Biotechnology, Santa Cruz, CA, USA), Bcl- ×L (Cell Signaling Technology) and γ-tubulina (Sigma, Saint Louis Missouri, USA).

### Cellular growth assays

XTT assays: The *in vitro* drug sensitivity in MSTO and NCI was assessed by Cell Proliferation kit (XTT), according to the manufacturer’s instructions. The assay is based on the cleavage of the yellow tetrazolium salt XTT to form an orange formazan dye by metabolic active cells. The drug was administered at doses and intervals as indicated. Absorbance was measured at 492 nm with a reference wavelength at 650 nm and the absorbance values of treated cells are presented as a percentage of the absorbance of dimethyl sulfoxide (DMSO) treated cells (CNTRL). All experimental points were quantified fivefold. Every single point was compared to their respective control with the same amount of DMSO. The anti-proliferative drug activity was assessed in a monolayer culture condition by plating cell lines in T25 flask. After 24 h, vehicle (DMSO) and exemestane were added at different concentrations for the time indicated in the experiment. The expansion of culture cell proliferation was quantified by manual cell counting. Experiments were repeated in triplicate and media values were calculated.

Colony formation assay: five hundred viable cells per well (treated with exemestane and CNTRL) were plated and allowed to grow in normal medium for 10 (MSTO and NCI) and14 (Met5A) days and then stained for 30 min at room temperature with a 6% glutaraldehyde, 0.5% crystal violet solution. Pictures were captured digitally and colonies were counted. All experiments were repeated at a minimum twice for each cell line.

### Wound healing assay

Cells (MSTO, NCI, Ist-Mes1, Ist-Mes2 and MPP89) grown to 95% confluence were seeded in 6-well tissue culture plates and wounded with a sterile 10-μL pipet tip to remove cells. Digital micrographs were taken after scratching and at the indicated times.

### Cyclic adenosine monophosphate (cAMP) assay

MPM cells (MSTO, NCI, Ist-Mes1, Ist-Mes2 and MPP89) were seeded into a T25 flask with phenol-red free DMEM/F12 for 24 h, then incubated in the presence or absence of exemestane for 30 min. The cAMP amount in the lysate was measured by ELISA according to the manufacturer’s instructions. This assay is based on the competitive binding technique. A monoclonal antibody specific for cAMP binds to the goat anti-mouse antibody coated onto the microplate. Following a wash to remove excess monoclonal antibody, cAMP present in a sample competes with a fixed amount of horseradish peroxidase (HRP)-labelled cAMP for sites on the monoclonal antibody. This is followed by another wash to remove excess conjugate and unbound sample. A substrate solution is added to the wells to determine the bound enzyme activity. The colour development is stopped and the absorbance is read at 450 nm. The intensity of the colour is inversely proportional to the concentration of cAMP in the sample.

### Flow cytometry

Cell cycle analyses cells were fixed in 70% ethanol and stored at -20°C over night. Fixed cells were treated with 1 mg/ml RNase A (cat. 12091021, Invitrogen) for 1 h at 37°C and DNA was stained with Propidium Iodide (Sigma). Samples were acquired with a Guava EasyCyte 8HT flow cytometer (Millipore). Cell cycle distribution is shown.

CD 44 analysis: The CD44 expression was evaluated by flow cytometry on the MSTO, NCI, Ist-Mes1, Ist-Mes2 and MPP89 MPM cell lines utilizing a FACSCanto flow cytometer (BD Biosciences, Franklin Lakes, NJ, USA) equipped with FACSDiva v6.1.3 data acquisition and analysis software (BD, San Jose, CA). Ten microL of the CD44-Fitc (BD Pharmingen) McAb was utilised to evaluate the percentage and mean intensity of fluorescence (MIF) of the MPM cell lines before and 24 hours after exemestane treatment. MPM single cell suspension was washed with phosphate buffered saline (PBS) pH 7.2–7.4, then spun at 1.500 rpm for 10 minutes, supernatant decanted, and incubated with the directly conjugated CD44 McAb utilizing the BD FACS Lyse and Wash Assistant according to the Duo-Lyse program (BD Biosciences, San Jose, CA, USA). Data was collected until the end of the aliquot was achieved. Data is presented as counts of positive cells and CD44 mean fluorescence intensity of total cell population in the sample analyzed.

### CD44 short interfering RNA (siRNA)

siRNA oligonucleotide targeting CD44 was transfected into MPM cells using lipofectamine 2000 following the manufacturer’s instructions using 200 nmol siRNA per 10 cm dish. Cells were incubated with siRNA for 5 hours and then left for 48 hours to achieve knockdown of CD44 protein as measured by immunoblot. Control cells were transfected with a scrambled siRNA oligonucleotide at matching concentration. Cells were then treated with vehicle or exemestane for 30 min and 24 hours and assayed for CD44, pCREB, pAKT and Bcl-xL by western blot.

### Western blot analysis

Briefly, 25–50 μg of proteins extracted as described previously [50] from cultured cells were separated by SDS-PAGE and transferred onto nitrocellulose membranes. Membranes were blocked and blotted with relevant antibodies. Horseradish peroxidase–conjugated secondary antibodies were detected by Enhanced ChemiLuminescence (ECL Amersham Biosciences). Goat anti mouse or rabbit IgG horseradish peroxidaseconjugated secondary antibodies (1:3.000) (Bio-Rad Laboratories; Hercules, CA, USA) were used.

### *In vivo* animal models

Female and male nude mice (6–8 weeks old; weight 18–25 g) were obtained from Charles River. Mice were housed in the animal facility of the Regina Elena National Cancer Institute for 2 weeks before each experiment; animals had *ad libitum* water and food. The Ethics Committee of the Cancer Institute approved all the experimental protocols that were carried out in accordance with Italian regulations and with the Guide for the Care and Use of Laboratory Animals. A mouse xenograft model of mesothelioma was created as described previously [51]. MSTO cell suspensions (2.5 × 10^6^) in 0,2 ml of complete medium were injected subcutaneously into the flank of CD1 nude mice (*n* = 12 (7 males and 5 females)/treatment group) and growth was measured twice weekly with calipers and calculated by the formula: 4/3 π (large diameter) × (small diameter)^2^. After the establishment of palpable lesions (average diameter >5 mm), mice were assigned to one of the following treatment groups: 1) Control, 2) Exemestane (8.25 mg/Kg, intraperitoneal (i.p.) 5 days a week). After testing the efficacy of exemestane alone, MSTO cell suspensions were injected subcutaneously into the flank of CD1 nude mice (*n* = 10 (5 males and 5 females)/treatment group) and mice were assigned to one of the following treatment groups 3) Cisplatin (3 mg/Kg i.p. once every 21 days) and Pemetrexed (150 mg/Kg i.p once every 21 days), 4) Exemestane (8.25 mg/Kg, i.p. 5 days a week) and Pemetrexed (150 mg/Kg i.p once every 21 days). A week before starting treatment in groups 3 and 4 an intramuscular dose of Vitamin B12 0.58 mg/kg was given. We chose the dose and the schedule of treatment by simulating those used in humans. Experimental groups were treated for 60 days. Mice were followed for tumor size, well being, and body weight and sacrificed 100 days after the start of treatment.

### Statistics

Cell culture–based assays were repeated at least 3 times; mean ± SD was calculated. Cell lines were examined separately. Differences in xenograft tumor size *in vivo* were assessed using a 2-tailed Student’s *t* test. Significance was set at P < 0.05.

## Abbreviations

MM: Malignant Mesotheliomas; MPM: Malignant Pleural Mesothelioma; EGFR: Epidermal Growth Factor Receptor; MAPK: Mitogen-Activated Protein Kinase; CYP19A1: Aromatase; cAMP: Cyclic adenosine monophosphate; CREB: cAMP response element-binding protein; PI3K: Phosphoinositide 3-kinases; GPCR: G-protein-coupled receptors; CNTRL: Control; DMSO: Dimethyl sulfoxide; PBS: Phosphate buffered saline; siRNA: Short Interfering RNA; ECL: Enhanced ChemiLuminescence; sd: Standard deviation.

## Competing interests

The authors declare that they have no competing interests.

## Authors' contribution

BN performed all cellular experiments. SG and GC performed animal studies. CM performed the siRNA assays. RS performed the cell cycle analysis by flow cytometry. SM performed the CD44 analysis by flow cytometry. IC supervised the experiments on CD44. RG creator of the study has provided critical input to the overall research direction and she wrote the paper with input from all co-authors. All authors read and approved the final manuscript.
